# Antioxidative Stress and Anti-Inflammatory Activity of Fucoidan Nanoparticles against Nephropathy of Streptozotocin-Induced Diabetes in Rats

**DOI:** 10.1155/2022/3405871

**Published:** 2022-05-31

**Authors:** Giftania Wardani, Jusak Nugraha, Mohd. Rais Mustafa, Sri Agus Sudjarwo

**Affiliations:** ^1^Doctoral Program of Medical Science, Faculty of Medicine, Universitas Airlangga, Surabaya, Indonesia; ^2^Program Study of Pharmacy, Faculty of Medicine, Hang Tuah University, Surabaya, Indonesia; ^3^Department of Clinical Pathology, Dr. Soetomo Hospital, Universitas Airlangga, Surabaya, Indonesia; ^4^Department of Pharmacology, Faculty of Medicine, University of Malaya, 50603 Kuala Lumpur, Malaysia; ^5^Department of Pharmacology, Faculty of Veterinary Medicine, Universitas Airlangga, Surabaya, Indonesia

## Abstract

Oxidative stress and inflammation have been shown to interact and have the role of importance in causing diabetic nephropathy complications. Fucoidan has a strong antioxidant and anti-inflammation effect, so the aim of this research was to evaluate the antioxidative stress and anti-inflammatory effect of fucoidan nanoparticles against nephropathy of streptozotocin-induced diabetes in rats. Fucoidan nanoparticles are characterized using dynamic light scattering (DLS) and scanning electron microscope (SEM). The rats were randomized into the control group (were given with aquadest), streptozotocin group (were injected with streptozotocin at a dose of 55 mg/kg BW i.p.), and fucoidan nanoparticle group (were given orally with fucoidan at doses 75, 150, and 300 mg/kg BW and then injected streptozotocin at a dose of 55 mg/kg BW i.p.). The blood was taken to evaluate the level of blood urea nitrogen (BUN) and creatinine. The kidney tissues were collected to measure malondialdehyde (MDA), interleukin-6 (IL-6), and tumor necrosis factor *α* (TNF-*α*) by ELISA; superoxide dismutase (SOD), and glutathione peroxidase (GPx) by immunohistochemical staining and histological observation by Hematoxylin & Eosin (H&E) staining. The DLS demonstrated that the fucoidan nanoparticle size was 330.6 ± 58.8 nm, and the SEM showed an irregular shape with a rough surface image. The administration of streptozotocin significantly increased BUN, creatinine, MDA, IL-6, and TNF-*α* levels, whereas expression of SOD and GPx decreased as compared with the control group (*p* < 0.05). The administration of fucoidan nanoparticles only at a dose of 300 mg/kg BW significantly decreases BUN, creatinine, MDA, IL-6, and TNF-*α* levels. However, fucoidan nanoparticles at a dose of 300 mg/kg BW significantly increase SOD and GPx expression as compared with the streptozotocin group (*p* < 0.05). The administration of streptozotocin caused the loss of normal kidney cell structure and necrosis, while treatment with fucoidan nanoparticles improved renal cell necrosis. It can be concluded that fucoidan nanoparticles are promising agents in terms of the protection afforded against streptozotocin-induced nephropathy through antioxidative stress by decreasing MDA and increasing SOD and GPx and through anti-inflammatory effect by decreasing levels of IL-6 and TNF-*α*.

## 1. Introduction

Hyperglycemia is the sign of diabetes mellitus (DM) that it is a very high prevalence and can cause death due to complications in several organs of the body. Hyperglycemia that lasts a long time can cause tissue damage and can cause various complications such as retinopathy, atherosclerosis, neuropathy, cardiomyopathy, and diabetic nephropathy [1, 2]. Diabetic nephropathy is a significant cause of chronic kidney disease and end-stage renal failure globally due to the presence of genetic susceptibility, glycometabolic disorders, changes in renal hemodynamics, oxidative stress, and inflammatory cytokines [3, 4]. Oxidative stress and inflammation have been shown to interact and have a pivotal role in causing diabetic nephropathy complications [5, 6].

Oxidative stress is a condition that occurs during an imbalance between the production of reactive oxygen species ((ROS) increasing (superoxide anions (O_2_^−^), hydroxyl radical (OH^−^), hydrogen peroxide (H_2_O_2_)), and antioxidant defense system (SOD, GPx, and catalase) decreasing [7, 8]. The increasing formation of ROS can cause diabetic complications, through (a) increased production of advanced glycation end products (AGEs), (b) pathway flux of polyol, (c) the hexosamine pathway overactivity of (d) increasing expression of the receptor for AGEs, and (e) protein kinase C isoforms activation [9, 10]. It has been reported that oxidative stress is involved in the pathogenesis of diabetic nephropathy. ROS can oxidize lipid components to produce MDA. The results of the MDA examination can be used as a biomarker for increased ROS production, which is an indicator of free radical damage under oxidative stress [11, 12].

On the other hand, cytokines of inflammatory such as IL-6 and TNF-*α* also cause impaired function and damaged kidneys in diabetes. In diabetes, renal cells (epithelial, mesangial, endothelial, and tubular cells) produce the cytokine of inflammatory IL-6 and TNF-*α*. Therefore, these inflammatory cytokines play a pivotal role and are involved in the progression of diabetic nephropathy complications [13]. It has been demonstrated that hyperglycemia causes the IL-6 and TNF-*α* increase; through the oxidative mechanism, research on diabetic patients has shown a significant association between IL-6, TNF-*α*, and diabetic nephropathy that can be used as indicators of diabetic nephropathy [5, 14, 15]. Thus, ingredients that can inhibit oxidative stress and inflammation are essential for the treatment and prevention of diabetic nephropathy.

The previous research showed that the presence of impaired function and a damaged kidney in a diabetic rat model of streptozotocin is the same as that of inhuman diabetic nephropathy [12, 16]. Streptozotocin also caused lower levels of SOD and GPx and higher MDA, IL-6, and TNF-*α* levels in the kidney tissues of a diabetic rat. Nephropathy in a diabetic rat model can be seen with an increase in BUN and creatinine in serum as a marker of impaired kidney function [17]. It was reported that streptozotocin can cause oxidative stress and inflammation, which can further damage the kidneys in diabetic rat model complications and eventually lead to nephropathy. Thus, agents that have antioxidant and anti-inflammation effects can be used to prevent nephropathy in diabetes [18, 19]. It has been reported that fucoidan is a natural product that has a strong antioxidant effect. Fucoidan derived from algae has been studied intensively during the last years regarding its antioxidant activities and therapeutic potential. Flucoidan also has pharmacological properties such as anti-inflammatory, anticancer, antibacterial, immunostimulant, antidiabetic, antiatherosclerosis, and antioxidant [20–22].

Recently, it has been demonstrated that nanobiotechnology has an essential role that is shown by the presence of synthesis of natural product nanoparticles. Therefore, natural product nanoparticles are seen as having opportunities in preventing and treating diseases, both in humans and animals. The synthesis of natural products based on nanoparticles when it is compared to purely natural products offers more improvement in drug stability, treatment efficacy, and penetration power [23–25].

From the explanation above, the aim of this research was to evaluate the antioxidative stress and anti-inflammation effect of fucoidan nanoparticles to protect kidney cells damaged in streptozotocin-induced diabetic rats.

## 2. Materials and Methods

### 2.1. Manufacturing of Fucoidan Nanoparticles by Ball Milling Methodology

The powder of fucoidan was milled using a high-energy ball equipped with an insulating sheath and a cooling machine. The mixture ratio of steel balls and fucoidan powders was around 20:1 by weight percent. The container is filled about a third of its capacity. During milling, the flask was rotated at a constant milling speed at 500 rpm for up to 5 h. The direction of rotation of the ball mill is changed every 30 minutes. The process of ball milling is conducted at a temperature of 27°C, and the temperature has maintained with the air conditioning system to prevent overheating.

SEM was used to evaluate the characteristics of morphology of the surface, including the shape, size, and topography of the fucoidan nanoparticles and then also carried out the identification particle size of fucoidan nanoparticles by DLS (Horiba LA 900, Japan).

### 2.2. Ethical Approval

We conducted all animal experiments based on the guidelines approved by the Animal Use Committee (Approval number: No.200/FK. UHT/V/2021), and all procedures of experiments have been agreed upon by the Committee of the Ethical Clearance for Research of preclinical, Faculty of Medicine, Hang Tuah University, Surabaya, Indonesia.

### 2.3. Experiment and Animals

Wistar male rats, which were healthy weighed 200–250 g and aged 2.5 to 3 months, were used in the study. These rats were obtained from the University of Airlangga, Surabaya, Indonesia. In this experiment, the rats were put in a plastic cage and placed in an air-conditioned room with the temperature maintained at 26 ± 2°C; in addition, the dark and light cycles were alternated for 12 hours. The rats for this experiment were given fed a standard commercial drinking water ad libitum.

### 2.4. Diabetic Model Rat

The rat fasted overnight and then was injected with streptozotocin at a dose of 55 mg/kg BW intraperitoneal (i.p.) that dissolved in citrate buffer (0.1 M; pH 4.5). Three days after streptozotocin injection, blood samples were taken through the lateral vein of the tail and tested for blood glucose levels by the glucometer (Accu-Check, Roche Diagnostics, Pvt., Ltd.). Rats with a level of glucose >250 mg/dL could be used as experimental animals.

### 2.5. Experimental Designs

Forty rats were randomized into the control group (rats were given aquadest), streptozotocin group (rats were injected with streptozotocin at a dose of 55 mg/kg BW i.p.), and fucoidan nanoparticles group (rats were injected with streptozotocin at a dose of 55 mg/kg BW and after 3 days and given fucoidan nanoparticles at doses of 75, 150, and 300 mg/kg BW orally once a day for 75 days). On day 75th of all groups of rats, blood was taken intracardially for examination of BUN and creatinine levels. The kidney was collected and fixed in 10% buffered formalin for observation of kidney damage in histological preparation. And the levels of MDA, IL-6, and TNF-*α* were measured by ELISA, and the expression of SOD and GPx were measured by immunohistochemical staining.

### 2.6. Measurement of Inflammatory Cytokines IL 6 and TNF in Diabetic Rat Kidneys

A total of 50 mg of kidney tissues were washed with 1% phosphate-buffered saline (PBS) five times until clean. The sample was pounded with a mortar and then was added 0.5 ml of sample buffer, and centrifuged at 10,000 rpm for 10 minutes. The supernatant was taken. Rat IL-6 ELISA kit PicoKine™ Boster was used to measure the Il-6 level. Similarly, TNF-*α* was also measured with Rat TNF-*α* ELISA kit PicoKine™ Boster, according to the manufacturer protocol. Place the sample in a standard microplate and then incubate at 37°C for 90 minutes. Add biotinylated antibody and incubate the plate at 37°C for 60 minutes and wash it three times with PBS 0.01 M. Add Avidin–Biotin Complex working solution and incubate the plate at 37°C for 30 minutes. Wash the plate with PBS 0.01 M. Add TMB color developing agent and incubate at 37°C for 20 minutes. Add 3,3′,5,5′-tetramethylbenzidine (TMB) stop solution and read the OD value on a 450 nm microplate reader. Furthermore, a standard curve is made between the values of OD to concentration so that we get the IL-6 or TNF-*α* concentration levels in pg/ml.

### 2.7. Measurement of MDA in Diabetic Rat Kidney Tissues

MDA was measured in the supernatant of homogenized kidney tissues using the thiobarbituric acid (TBA) technique, which predicts MDA production using a TBARS assay kit (Cayman Chemical Company, Ann Arbor, MI, USA). The absorbance coefficient of the MDA-TBA complex was used to assess the level of MDA, which was measured at 532 nm on a microplate reader. The extent of lipid peroxidation was quantified by estimating the MDA concentration. The results of MDA are expressed in nanomoles per milligram of tissue.

### 2.8. Immunohistochemical Staining of Antioxidant Enzymes in Kidney Tissues

Immunohistochemical staining was utilized to observe SOD and GPx expression. Kidney tissue slices of 4 *μ*m were deparaffinized and was added hydrogen peroxide at 37°C for 10 minutes to inhibit endogenous peroxide. Then, 10% normal sheep serum was given in Tris-buffered salt solution at 37°C for 30 minutes. Furthermore, incubated overnight at 4°C with anti-rat anti-SOD monoclonal (1:100; ab8376; Abcam, Cambridge, MA, USA) or anti-rat anti-GPx monoclonal (1:100; sc8008, Santa Cruz Biotechnology) antibodies. After that, We washed three times with PBS and incubated with a secondary antibody from the UltraVision Quanto Detection System HRP DAB (Thermo Fisher Scientific, Waltham, MA, USA) for 30 minutes at room temperature, and with 3.3′ diaminobenzidine (DAB) color reagent. Immunohistochemical expressions were observed by microscopy and semiquantified by Image-Pro Plus 6.0 software. The integrated optical density (IOD) of each photo was collected. Images were measured by immunoreactive area (IA) in *μ*m^2^ and IOD. The staining intensity (SI) for each image was calculated as SI = IOD/IA and the mean with standard deviation.

### 2.9. Histopathological Examination

Rats were sacrificed, and their kidneys were collected and fixed in 10% buffered formalin solution, dehydrated in ethanol, and embedded in paraffin. Kidney tissue sectioned at 5 *μ*m was stained with hematoxylin and eosin. The sections were examined under a microscope for the presence of indicators of cellular damage such as tubular necrosis and renal tubular degeneration.

### 2.10. Biochemistry Evaluation of Creatinine and BUN

Blood samples were collected for the estimation of serum creatinine and BUN using commercial enzymatic kits (Reckon Diagnostics) according to the supplier's specifications and were determined by spectrophotometry (ILab Aries; Instrumentation Laboratory, Milan, Italy) using commercial kits (Instrumentation Laboratory).

### 2.11. Statistical Analysis

The data were presented in the form of means ± standard deviation. The one-way analysis of variance (ANOVA) is used to analyze the data and will be continued with the LSD test through the application of SPSS 17.0 (SPSS Inc., Chicago, USA).

## 3. Results

### 3.1. Scanning Electron Microscope for Characterization of Fucoidan Nanoparticles

The ball milling was used in the preparation of fucoidan. SEM images showing the morphology of fucoidan nanoparticles, rough surface, and shape irregular is presented in Figure 1.

### 3.2. Dynamic Light Scattering Is Used in the Characterization of Fucoidan Nanoparticles

As shown in Figure 2, the average particle size of the fucoidan nanoparticles produced by DLS was 330.6 ± 58.8 nm.

### 3.3. Effects of Fucoidan Nanoparticles on MDA Level of the Kidney Tissue of Streptozotocin-Induced Diabetic Rats

The MDA production can be used as a biomarker for increased ROS production, which is an indicator of kidney cell damage under oxidative stress. The results of the study of kidney MDA levels are presented in Table 1. MDA is the production of lipid peroxidation whose levels increase in oxidative stress. The administration of streptozotocin significantly increased MDA levels in kidney tissue compared to the control group (*p* < 0.05). In diabetic nephropathy, rats treated with fucoidan nanoparticles significantly reduced MDA levels at a dose of 300 mg/kg BW but not at a dose of 75 mg/kg BW and 150 mg/kg BW (*p* < 0.05).

### 3.4. Effect of Fucoidan Nanoparticles on SOD Expression of the Kidney Tissue of Streptozotocin-Induced Diabetic Rats

The role of SOD as a first-line antioxidant defense is important and indispensable to prevent kidney cell damage due to ROS. The expression of SOD in kidney tissue is presented in Figure 3. The administration of streptozotocin significantly decreased the expression of SOD in kidney tissue compared to the control group (*p* < 0.05), However, dose-dependent treatment with fucoidan nanoparticles could increase SOD expression in kidney tissue and only at a dose of 300 mg/kg BW could significantly increase SOD (Figure 3) expression compared to the streptozotocin group (*p* < 0.05).

### 3.5. Effect of Fucoidan Nanoparticles on GPx Expression of the Kidney Tissue of Streptozotocin-Induced Diabetic Rats

Antioxidant enzymes such as GPx have a pivotal role in protecting oxidative cell injury caused by ROS. The expression of GPx in kidney tissue is presented in Figure 4. The administration of streptozotocin significantly decreased the expression of GPx in kidney tissue compared to the control group (*p* < 0.05). However, dose-dependent treatment with fucoidan nanoparticles could increase GPx expression in kidney tissue and only at a dose of 300 mg/kg BW could significantly increase GPx (Figure 4) expression compared to the streptozotocin group (*p* < 0.05).

### 3.6. Effect of Fucoidan Nanoparticles on Inflammatory Cytokines of the Kidney Tissue of Streptozotocin-Induced Diabetic Rats

Cytokines of inflammatory such as IL-6 and TNF-*α* play a pivotal role in kidney damage that can be used as indicators of diabetic nephropathy. To prove that fucoidan nanoparticles are involved in regulating inflammatory cytokines in streptozotocin-induced kidney damage in diabetic rats, we measured the inflammatory cytokines level of IL-6 and TNF-*α*. As presented in Table 2, the administration of streptozotocin significantly increased the level of IL-6 and TNF-*α* in kidney tissue compared to the control group (*p* < 0.05). However, dose-dependent treatment with fucoidan nanoparticles could decrease the levels of IL-6 and TNF-*α* in kidney tissue and only at a dose of 300 mg/kg BW could significantly decrease the level of IL-6 and TNF-*α* compared to the streptozotocin group (*p* < 0.05).

### 3.7. Effect of Fucoidan Nanoparticles on BUN and Creatinine Levels in the Serum of Streptozotocin-Induced Diabetic Rats

The diagnosis of kidney damage is usually based on measurements of BUN and serum creatinine. The effects of fucoidan nanoparticles on the level of BUN and Creatinine in the serum of diabetic rats are presented in Table 3. The administration of streptozotocin significantly increased BUN and creatinine levels in serum compared with the control group (*p* < 0.05). This result indicates that streptozotocin could cause kidney cells damaged in rats. However, dose-dependent treatment with fucoidan nanoparticles could decrease the level of BUN and creatinine in kidney tissue and only at a dose of 300 mg/kg BW could significantly decrease the level of IL-6 and TNF-*α* compared to the streptozotocin group (*p* < 0.05).

### 3.8. Effect of Fucoidan Nanoparticles on the Structural Changes of the Kidney Tissue of Streptozotocin-Induced Diabetic Rats

To prove the nephroprotective of fucoidan nanoparticles, we conducted histopathological examination of streptozotocin-induced diabetic nephropathy rats. Light microscopic examination revealed that the control group exhibited normal structure of the kidney. The administration of streptozotocin can cause morphological irregularities, several tubular degenerations, and tubular necrosis (Figure 5). The treatment with fucoidan nanoparticles could inhibit tubular necrosis and protect the normal structure of the kidney.

## 4. Discussion

Hyperglycemia is one of the signs of diabetes mellitus (DM), which can produce excessive ROS in the body and lead to the production of inflammatory cytokines increasing and accelerating kidney cell damage in diabetes. Interaction of oxidative stress and inflammation has a very pivotal role in the pathogenesis and progress of kidney damage in diabetes, which is called nephropathy [3, 4].

In diabetes, excessive ROS production can reduce antioxidant defenses, leading to the oxidation of proteins, DNA, and lipids, resulting in diabetic nephropathy [2, 26]. In addition, hyperglycemia is vulnerable to oxidative stress-induced cell damage due to inhibited antioxidant ability through glycation of scavenging enzymes, such as SOD and GPx. It is also due to the interaction of glucose with proteins that AGEs are formed, which block receptors and inactivate enzymes [1, 2].

Since oxidative stress and inflammation in the rat model of diabetes caused by streptozotocin have an important role in the progress of diabetic nephropathy, so it is necessary to evaluate several oxidative stress and inflammatory cytokine parameters such as MDA, SOD, GPx, IL-6, and TNF-*α* [3, 4]. Streptozotocin can interfere with the function of the beta cells of the islets of Langerhans resulting in inhibition of insulin release, which in turn leads to hyperglycemia and diabetes complications such as diabetic nephropathy. The aim of the research was to evaluate the potency of antioxidative stress and anti-inflammatory effect of fucoidan nanoparticles to protect from STZ-induced diabetic nephropathy in rats.

Drug nanotechnology can be used to improve biodistribution, specificity, sensitivity, and reduce pharmacological toxicity [23, 24]. Furthermore, the milling process is carried out to make fucoidan nanoparticles. And the results of fucoidan nanoparticles from this study indicate that the particle size of 330.6 ± 58.8 nm is expected to the effectiveness of its antioxidative stress and anti-inflammatory increase.

In the present research, streptozotocin-induced diabetic nephropathy showed that MDA levels increased; however, SOD and GPx expression reduced significantly (*p* < 0.05) compared to the control group. The administration of fucoidan nanoparticles was only at a dose of 300 mg/kg b.w. decreased MDA levels and increased SOD and GPx expression significantly (*p* < 0.05) as compared with the streptozotocin-induced diabetic nephropathy. MDA is a lipid peroxidation product that can be used as a marker of increased ROS formation in tissue damage. Streptozotocin is known to increase MDA levels in tissues of various organs including kidneys [27]. These results suggest that the administration of fucoidan nanoparticles in a dose-dependent manner inhibits oxidative stress that may protect the development of nephropathy in diabetic rats. These results are in agreement with the previous report that the scavenging of ROS by fucoidan may be partially related to the increased activity of antioxidant enzymes. The free radical scavenging activity of fucoidan can be attributed to the presence of ^−^OH groups in the polysaccharide unit of fucoidan that can react with hydroxyl free radicals (^*∗*^OH) in the test of hydroxyl radical assay. Cell possesses an intricate network of defense mechanisms, including antioxidant compounds such as GSH and antioxidant enzymes such as superoxide dismutase, catalase, and glutathione peroxidase to neutralize excessive ROS accumulation. Oxidative stress in hyperglycemia is a key role in the progression of kidney injury, which relates to diabetic nephropathy. Hyperglycemia is recognized to induce oxidative stress with an imbalance between decreased antioxidant defense and increased ROS production. The administration of antioxidants fucoidan nanoparticles can improve kidney function by preventing oxidative tissue damage in diabetic nephropathy. The same result, the administration of exogenous antioxidants such as *Syzygium aromaticum*, *Black mulberry* fruit, and *Heteroxenia ghardaqensis* can inhibit ROS formation by scavenging the intracellular ROS that has been formed [17, 18, 28].

On the other hand, inflammatory cytokines have also been associated with nephropathy in diabetic patients. Our research describes that inflammatory cytokines IL-6 and TNF-*α* levels in kidney tissue are significantly increased in streptozotocin-induced diabetic nephropathy rats, indicating that these rats have kidney damage. We demonstrated that fucoidan nanoparticles at a dose of 300 mg/kg BW but not at a dose of 75 mg/kg BW and 150 mg/Kg BW significantly reduced IL-6 and TNF-*α* levels in the kidney tissue of diabetic rats. This result suggested that fucoidan nanoparticles inhibit the inflammation effect in protecting kidney damage in diabetic rats. The most discussed possible mechanism of anti-inflammatory effect of fucoidan is the downregulation of MAPK and NF-*κ*B signaling pathway and the following decrease in the production of inflammatory cytokine IL-6 and TNF-*α*. Inflammation has also an important role in the occurrence of nephropathy in diabetes. Hyperglycemia may also cause diabetic nephropathy through ROS activation, further accelerating the production of inflammatory cytokines such as IL-6 and TNF-*α*, leading to diabetic nephropathy [4, 5]. Previous studies have also shown that administration of exogenous antioxidants can inhibit diabetic nephropathy due to inhibition of oxidative stress, resulting in a decrease in the production of inflammatory cytokines such as IL-6 and TNF-*α* [3, 6].

In the results, we also showed that kidney functional impairment in streptozotocin-induced diabetic nephropathy was evidenced by the increased levels of biochemical markers such as BUN and creatinine, which were significantly higher as compared with the control group. The administration of fucoidan nanoparticles at a dose of 300 mg/kg BW but not at doses of 75 mg/kg BW and 150 mg/Kg BW significantly reduced BUN and creatinine levels in the kidney cell damage of diabetic rats. Streptozotocin-induced nephropathy is characterized by elevated serum BUN and creatinine levels that are associated with increased ROS formation in oxidative stress [15]. The ability of antioxidants to remove ROS has been demonstrated to be an important role in contributing to nephroprotective efficacy. The administration of fucoidan nanoparticle significantly decreases streptozotocin-induced kidney cell damage, which is related to reduced creatinine and BUN serum levels, suggesting that fucoidan nanoparticles have the ability to inhibit kidney cell damage caused by streptozotocin. These results are in agreement with previous research that the antioxidant enzyme has the ability to inhibit streptozotocin-induced nephropathy as shown by decreased levels of BUN and creatinine in serum [17]. In the present research, the fucoidan nanoparticles can protect against streptozotocin-induced kidney damage. This result is the first research to report the inhibition of streptozotocin-induced kidney injury by fucoidan nanoparticles in rats significantly. Kidney function was also increased, demonstrated by a decrease in BUN and creatinine, and accompanied by inhibition of kidney oxidative stress, which was indicated by a decrease in kidney MDA levels, an increase in antioxidants expression (SOD and GPx activities), and an increase in inflammatory cytokines (IL-6 and TNF-*α*). Fucoidan nanoparticles inhibit kidney cell damage induced by streptozotocin, as evidenced by reduced BUN and creatinine levels in kidney tissue; furthermore, the histological observation clearly indicates that necrosis in the tubular induced by streptozotocin was remarkably decreased by the administration of fucoidan nanoparticle. This study shows that fucoidan nanoparticles have nephroprotective activity through antioxidants and anti-inflammatory. Therefore, it is hoped that fucoidan nanoparticles can be used to help people with diabetes prevent complications such as retinopathy, nephropathy, atherosclerosis, and cardiomyopathy. Furthermore, it is necessary to investigate the antiapoptotic role of fucoidan nanoparticles in diabetic nephropathy.

## 5. Conclusion

The nephroprotection of fucoidan nanoparticles appears to be related to the antioxidative stress that suppresses MDA and increases SOD and GPx expression and the anti-inflammatory effect that decreases IL-6 and TNF-*α*, which can further decrease BUN and creatinine levels in diabetic nephropathy.

## Figures and Tables

**Figure 1:** Scanning electron microscope images of fucoidan nanoparticles.

**Figure 2:** Size distribution of fucoidan nanoparticles by dynamic light scattering.

**Figure 3:** Photomicrographs of immunohistochemical staining of SOD expression of rat kidney tissue: (a) SOD expression in rat kidneys from the control group (A), streptozotocin group (B), and the fucoidan nanoparticle group with a dose of 75 mg/kg BW (C), 150 mg/kg BW (D), and 300 mg/kg BW (E) and (b) IOD/*µ*m^2^ shows SOD expression in semiquantitative evaluation (400x).

**Figure 4:** Photomicrographs of immunohistochemical staining of GPx expression of rat kidney tissue: (a) GPx expression in the rat kidney from the control group (A), streptozotocin group (B), and the fucoidan nanoparticle group with a dose of 75 mg/kg BW (C), 150 mg/kg BW (D), and 300 mg/kg BW (E) and (b) IOD/*µ*m^2^ shows GPx expression for semiquantitative evaluation (400x).

**Figure 5:** Photomicrographs of H&E staining of rat kidney tissue. The control group showed normal morphology in the kidney (a). The necrosis (black arrows) is found in the streptozotocin group (b). The treatment of fucoidan nanoparticles with 75 mg/kg BW and 150 mg/kg BW given to rats still indicated the presence of mild necrotic (c, d), while the treatment of nanoparticles of fucoidan 300 mg/kg showed the presence of regeneration in damaged kidney cells (e) (H&E, 400x).

**Table 1:** Effect of fucoidan nanoparticle on MDA levels of kidney tissues of streptozotocin-induced diabetic rat.

Group	Means ± SD
	MDA (nmol/mg)
Control group	2.24^a^ ± 0.28
Streptozotocin group	6.09^b^ ± 0.46
Fucoidan nano, 75 mg/kg BW	5.78^b^ ± 0.65
Fucoidan nano, 150 mg/kg BW	4.61^bc^ ± 0.53
Fucoidan nano, 300 mg/kg BW	3.82^cd^ ± 0.39

The different superscripts in each column show significant difference between the means (*p* < 0.05).

**Table 2:** Effect of fucoidan nanoparticles on IL-6 and TNF-*α* levels in the kidney tissue of streptozotocin-induced diabetic rats.

Group	Means ± SD	
	IL-6 (pg/mg protein)	TNF-*α* (pg/mg protein)
Control group	35.4^a^ ± 4.2	41.2^a^ ± 5.3
Streptozotocin group	89.3^b^ ± 7.3	107.6^b^ ± 9.2
Fucoidan nano, 75 mg/kg BW	92.8^b^ ± 8.5	104.3^b^ ± 7.8
Fucoidan nano, 150 mg/kg BW	83.6^b^ ± 6.9	98.7^b^ ± 6.2
Fucoidan nano, 300 mg/kg BW	48.1^c^ ± 4.3	65.8^c^ ± 6.7

The different superscripts in each column show significant difference between the means (*p* < 0.05).

**Table 3:** Effect of fucoidan nanoparticle on BUN and creatinine level in the serum of streptozotocin-induced diabetic rats.

Group	Means ± SD	
	BUN (mmol/L)	Creatinine (mmol/L)
Control group	9.3^a^ ± 3.21	32.1^a^ ± 4.18
Streptozotocin group	21.2^b^ ± 5.32	51.4^b^ ± 6.24
Fucoidan nano, 75 mg/kg BW	22.4^b^ ± 4.62	54.7^b^ ± 5.99
Fucoidan nano, 150 mg/kg BW	18.5^b^ ± 4.76	49.5^b^ ± 6.81
Fucoidan nano, 300 mg/kg BW	12.1^c^ ± 3.58	39.3^c^ ± 4.73

The different superscripts in each column show significant difference between the means (*p* < 0.05).

## Data Availability

The data used to support the findings of this research are included within the article.
